# An Assessment of Accessibility and Usability of Saudi Online FinTech Services for People with Disabilities

**DOI:** 10.1155/2022/8610844

**Published:** 2022-09-26

**Authors:** Redhwan Nour

**Affiliations:** Department of Computer Science, College of Computer Science and Engineering, Taibah University, Medina 42353, Saudi Arabia

## Abstract

Innovations in financial services have given rise to Financial Technology (FinTech) as a disruptive technology which is now shaping the future of the financial sector through services like crowdfunding, peer-to-peer loans, and alternative underwriting platforms. Given the status of the web as a vital information resource, accessible and usable online FinTech services can aid people with disabilities in taking full advantage of the presented financial services to support them in basic needs like accessing high-quality care. This study set out to analyze the accessibility and usability of 32 Saudi FinTech websites by means of various automated tools and manual inspection. The results revealed the investigated websites to have a significant number of accessibility and usability problems that cause prejudice against disabled individuals and foster an overall poor user experience. Thus, more work is needed to disseminate knowledge about the importance of developing suitable FinTech websites and services to assist disabled people.

## 1. Introduction

Emerging technologies have contributed greatly to new innovations in banking and the financial services sector, such as financial technology, abbreviated FinTech. In the words of the Financial Stability Board (FSB), FinTech is “Technology-enabled innovation in financial services that could result in new business models, applications, processes, or products with an associated material effect on the provision of financial services” [1]. Meanwhile, Schueffel describes it as “a new financial industry that applies technology to improve financial activities” [2]. While the above differ in their particulars and may not be fully comprehensive definitions, both agree on FinTech providing a means to improve financial service delivery to consumers. Distinct from the legacy infrastructure associated with banks, FinTech is centered on new developments and technologies such as artificial intelligence, big data, and cloud computing, and on achieving a seamless customer experience that is convenient, accessible, functional, and personalized.

FinTech originated with money transfers, crowdfunding, mobile payments, and peer-to-peer loans, and the scope of its activities has since broadened to include the more recent developments of blockchain, cryptocurrencies, and robo-investing [3]. The benefits FinTech firms offer to customers thus span numerous domains, from payments and lending to private fundraising and finance, banking activities and insurance to capital market access and treasury management, and more besides [4]. In expediting processes that historically required days, weeks, or even months to conduct, such as obtaining a credit score report or transferring money internationally, FinTech facilitates the access of diverse individuals to financial services. For example, online services enable consumers to use a digital health wallet, access health lending services, or choose from different health plans and benefits, in addition to navigating financially complex tasks such as loan or mortgage applications without need for any interaction whatsoever with an actual live person. Rather than meeting with a financial expert face-to-face or over the phone, clients can peruse options online or even take guidance from a chatbot.

This rapid development and innovation in payment methods, insurance products, care delivery services, and other areas has created tremendous opportunities to develop FinTech and healthcare solutions that aid people with disabilities. FinTech websites are thus a key starting point through which users engage with and benefit from FinTech services. As such, the ease of use and accessibility of these websites are critical factors in extending FinTech services to more diverse groups and engaging and retaining users. The accessibility of a website concerns user perception, understanding, navigation, interaction, and contribution, including compatibility of the site with different devices such as PCs and mobile phones [5]; meanwhile, usability concerns the website design and whether it is effective, efficient, and satisfying to the user [6]. For a website to be most effective, accessibility and usability should both be addressed during its design and development [7].

Designing and developing an accessible site requires accommodating all manner of disabilities that can affect a user's web access; in addition to visual disabilities, these include physical, auditory, speech, cognitive, and neurological disabilities, each of which imposes functional limitations. Such disabilities may be congenital, or may result from disease, an accident, or aging. In addition, different users face different challenges in different degrees, though some may share disabilities [8].

The Web Content Accessibility Guidelines (WCAG) represent a global standard intended to increase accessibility of online content for disabled individuals. Two versions have thus far been developed by the World Wide Web Consortium (W3C): WCAG 2.0 (from 2008) and WCAG 2.1 (from 2018). The newer version includes all requirements stipulated in the older, thus any website conforming to WCAG 2.1 is backwards-compatible with 2.0 [9]. The guidance laid out by the current standard includes 4 principles, 13 guidelines, and 78 Success Criteria (SC), of which 61 were inherited from WCAG 2.0 and 17 were introduced to address mobile accessibility and users having low vision, cognitive disabilities, or learning disabilities [10].

The core of the accessibility guidelines is encapsulated in the acronym “POUR”, which corresponds to the four principles. That is, an accessible website is *Perceivable*, meaning the content and user interface can be perceived regardless of a user's sensory abilities and means of access; it is *Operable*, meaning multiple modalities can be used to interact with the user interface and navigate the site; it is *Understandable*, meaning the site content and the purpose of its interface elements can be comprehended by users; and it is *Robust*, meaning the site functions reliably when accessed by diverse technologies, including assistive agents [10].

The SC represent specific aspects of compliance, and are divided into three levels: A, representing basic conformance with web accessibility requirements; AA, in which significant barriers have been addressed; and AAA, the highest degree of conformance but also the most difficult to achieve. Notably, these levels are cumulative: achieving level AA conformance indicates the stipulations of level A are also met [11].

The accessibility of a site can be tested by multiple means, including an initial check, manual evaluation (by a general user or an expert), and automated utilities [12]. A tool-based audit to determine accessibility conformance and provide a report on violations can address some limitations of other methods, such as the cost of an expert assessment [13] or difficulties in recruiting disabled individuals for testing [14]. According to a listing compiled by the W3C, over one hundred accessibility assessment tools have been developed [15], each offering a distinct set of features and functionalities and supporting the needs of different audiences such as designers, developers, and end users.

If a website has poor usability, users may have difficulty acquiring the information they need from it [16]. Conversely, a website with high usability is positively regarded and engenders in users greater degrees of satisfaction, trust, and even loyalty. Tools analyzing web usability do so through several steps, evaluating efficiency, effectiveness, and user satisfaction. Among the metrics used to assess usability include the size, load time, and holistic performance of a page, as speed of loading factors prominently in user experience. The number of broken links is another prominent usability metric, as broken links impede page indexing by search engine crawlers. Moreover, broken links redirect visitors to error pages, which negatively affect user experience. A third measure is the mobile-friendliness of a website. Sites that are not mobile-friendly may require users to zoom in just to read the content, which can cause frustration [17].

Having a search function available on a website is also important for both usability and accessibility [18]. In particular, search functions that retrieve content based on specific words or phrases allow the user to bypass needing to understand a website's structure and quickly find the content they require, especially on large sites. Providing multilingual content is also important, as site users may include nonnative residents who are not proficient in the country's predominant language. Thus, it must be feasible for the website to be switched into a language such users can readily understand. Accordingly, the SC 3.1.1 [19] and 3.1.2 [20] are aimed at ensuring user agents which convert text into synthetic speech are able to accurately deliver content provided in multiple languages.

By designing a FinTech website with due consideration of accessibility and usability, barriers are removed that might hinder disabled people from making use of the website, allowing anyone to access the offered services irrespective of their specific circumstances. Moreover, having a highly usable website that can be accessed in diverse ways promotes user satisfaction. Accordingly, developers of FinTech websites should endeavor to assure equal access of all users to the services their websites provide.

Among the goals of the Saudi Arabia Vision 2030 is reinforcing economic and investment activities, which has led to the National Digital Transformation Unit (NDU) being developed. This unit aims for “The Kingdom of Saudi Arabia to become a leading example of providing digital services centered on the citizen, resident, visitor, government agencies and the private sector” [21]. The Financial Sector Development Program (FSDP) is another initiative with the goal of enhancing innovation and competition by attracting key players in the field, aiming to have 525 FinTech companies functioning within the Kingdom by 2030 [22].

The Saudi Central Bank (SAMA) and the Capital Market Authority (CMA) serve to regulate FinTech companies in the Kingdom. In particular, SAMA gives approval for companies involved in open banking services, digital saving associations, crowdfunding platforms, and related domains, while CMA concentrates on robo-advisory, social trading, and distribution platforms for investments and real estate funds. In 2018, these regulators together launched the nonprofit FinTech Saudi [4], a cluster intended to catalyze development of the Kingdom as an innovative hub of financial services technologies and home to a FinTech ecosystem that is both thriving and responsible. Several initiatives have subsequently been put forth promoting development of the infrastructure needed to grow the FinTech industry, building capabilities, and talent, and to otherwise support entrepreneurs in this area regardless of their stage of development; these include an accelerator program, internships, tours, and a podcast.

In light of the above, this study is aimed at investigating and assessing the accessibility and usability of 32 websites belonging to Saudi FinTech companies, particularly those having received approval from the CMA and SAMA. Both automated tools and manual inspection were utilized to highlight accessibility and usability problems with the evaluated sites.

The rest of this paper is organized as follows: Section II summarizes related literature; Section III highlights the research method used; Section IV presents the accessibility and usability evaluation results; Section V discusses those results; and Section VI presents the conclusion of the study.

## 2. Related Work

There is a dearth of research that focuses on usable access to FinTech websites. However, online banking services have previously been reviewed and can be considered as falling under the umbrella of FinTech services. In a study examining the accessibility and usability of ten Nigerian banks [23], tool-based analyses revealed all the tested websites to harbor accessibility issues, of which failure to provide alternative text was the most frequent. Another common issue was slow user experience due to insufficient performance optimization. In addition, while 70% of tested websites were compatible with mobile view, all harbored broken links that impacted site usability.

Similarly, Akgül [24] evaluated 32 Turkish banking websites of various types (state-owned, privately-owned, foreign, etc.) and determined the majority to have significant accessibility errors, the most prevalent of which was a failure to supply text equivalents for every nontext element. Furthermore, the websites frequently had broken links; the smallest proportion of sites having broken links was found among privately-owned banks, at 75% of such sites.

Yanusha et al. [25] employed both experience and tool evaluation methods. They identified a need to give greater attention to speed of loading, mobile friendliness, and adherence to standards, and furthermore that customer expectations for all examined aspects of usability were not well-satisfied. Indeed, a separate survey of 162 blind users regarding their experiences with banking and finance websites or apps [26] found respondents to prefer using web banking services over physically visiting bank locations, yet they also reported banking websites to have accessibility problems pertaining to headers, alternative text, clear labels, timed content, and navigation. In addition, participant responses highlighted difficulties associated with CAPTCHA (Completely Automated Public Turing test to tell Computers and Humans Apart), including lack of audio options, inaccessibility of the buttons to activate audio CAPTCHA, and the audio CAPTCHA being itself unusable.

Pham et al. [27] likewise evaluated the accessibility of 18 websites belonging to the largest banks in the US and found that several did not fully comply with accessibility standards, identifying a total of 72 accessibility violations. The author concluded by suggesting that if banks want to offset reductions in physical banking accessibility, it they need to better attend to online baking accessibility.

Another study applied an automatic tool to evaluate accessibility for the homepages of 48 banking websites in India [28]. Again, no site was found to be perfectly accessible for those with disabilities, and there was no difference between public and private sector bank websites in terms of overall degree of accessibility compliance. Prominent accessibility issues for these sites included nontext content, link purpose (in context), and failure to identify the language of a page. Finally, ELISA [29] performed a similar assessment of 79 Tanzanian e-government websites using multiple tools. All the websites harbored broken links, a majority required an extended loading time for their main page, and 44% had page sizes higher than recommended, all of which contribute to a poor user experience. In addition, all websites returned accessibility errors related to the lack of an “alternative text” attribute on images and associated labels on form controls.

## 3. Method

### 3.1. Selected Websites

This study is aimed at evaluating Saudi FinTech company websites. It was decided to exclude banking websites as “FinTech” usually assumes a shift from traditional financial services to more modern and innovative ones. The inclusion criteria required that companies be authorized by the SAMA Sandbox or CMA FinTech Lab [30, 31]. In total, 32 websites (10 SAMA, 22 CMA) were analyzed in June and July 2022. Specifically, the Arabic version of each website's homepage was evaluated, except for the Wethaq website, which did not have an Arabic version and so the English version was used.

### 3.2. Assessment Tools

Three online web accessibility evaluation tools were employed: MAUVE++ [32], Siteimprove [33], and WAVE [34]. These tools have seen wide use in the literature [35–40] and all of them are listed by the W3C as appropriate for evaluation against the WCAG 2.1 guidelines [15]. More than one tool was utilized so that the assessment would benefit from more features and functionality and the limitations of each tool might be offset [41]. MAUVE++ supports validation for both individual pages and multiple pages, and produces reports in several different formats and tailored for distinct audiences. The Google Chrome extension Siteimprove similarly identifies accessibility issues and explains them, gives intuitive feedback in a visual manner, and finally offers suggestions for resolving the issues. WAVE also provides visual feedback, specifically in categorizing identified issues: problems with accessibility and contrast are shown in red, those that require manual intervention in yellow, and features and areas to be improved in green.

In addition, usability measurements were assessed with Pingdom [42], which tests website performance, load time, and page size, and with Dead Link Checker, which checks for broken links [43]. Mobile and tablet view compatibility was examined using the Google mobile friendly test tool [44]. Finally, a manual inspection was incorporated to check the availability of search functions and language options. All of the abovementioned tools and the manual method have been previously used in several studies [39, 45–48].

### 3.3. Procedure

First, the accessibility of a total of 32 homepages belonging to Saudi FinTech company websites was evaluated using three tools: WAVE, Siteimprove, and MAUVE++. All three conformance levels of WCAG 2.1 were evaluated, and any errors detected were manually analyzed. Second, usability testing was conducted with the Pingdom tool, in which each website's URL was entered and the “test from” option set to Asia-Japan and Tokyo. The resulting scores concerning page size, load time, overall performance, and website grade were then recorded. Dead Link Checker tallied broken links on each homepage and throughout each website. The Google mobile friendly test was applied to check friendless of the sites in regard to mobile view and report any usability problems. Finally, each website was manually checked for the inclusion of the search feature and language options. The evaluation took place in June and July 2022, and focused on the Arabic version of each homepage.

## 4. Results

### 4.1. Accessibility Analysis

The results of the assessment are presented in Table 1. Across all 32 FinTech homepages and all three accessibility tools, a total of 10766 violations were identified. MAUVE++ reported 78% of all errors, while the other two each reported 11%. The website with the greatest number of errors was the Rabet homepage with 2298 errors, while the least were obtained for MAKASSB with only 14 problems. Only three websites (Sahem, Dinar, Emkan) were reported by at least one tool as having no errors. However, no website was passed by all tools. Notably, the information for Yaqeen's website could not be retrieved by MAUVE++, and a validation error message consistently appeared.

Figure 1 highlights the most frequent errors reported by each tool and their corresponding percentages. MAUVE++ returned the highest number at 26, Siteimprove the second most at 21, and WAVE the least at only 12. Of the violations identified by MAUVE++, around 63% belonged to just three errors: “Using ARIA landmarks to identify regions of a page” (level A), “Specifying alignment either to the left OR right in CSS” (level AAA), and “Using percent, em units or named font sizes” (level AA). These three errors affected over 50% of tested websites. In fact, “Using ARIA landmarks to identify regions of a page” was the single most prevalent error, identified on 28 websites. All three of these errors are associated with the perceivable principle.

Siteimprove similarly reported just five types of errors, which encompassed more than 66% of all violations it identified. Two of those related to basic accessibility requirements (level A): “Image without a text alternative” and “Link without a text alternative”; one to intermediate requirements (level AA): “Color contrast is not sufficient”; and the remaining two to the highest guidelines (level AAA): “Font size is fixed” and “Line height is below minimum value”. Of those, “Link without a text alternative” comes under the operable principle, while the other four are linked to the perceivable principle.

The WAVE tool found two errors to constitute over 60% of all violations it detected both at the lowest level of conformance (level A): “Very low contrast” and “Missing alternative text”. Each of these errors was reported in half of the selected websites. Similar to the findings of the other tools, both of these errors belong to the perceivable principle.

### 4.2. Usability Analysis

As shown in Table 2, only four websites (13%) achieved excellent results in terms of performance; another three showed good performance, while the remaining received average and below average scores (average being 76). In fact, 18 websites (58%) scored below average, indicating some issues in performance. Moreover, 21 websites (68%) had page sizes exceeding 2 MB, where the size recommended by Google is less than 500 KB [49]. Additionally, 28 websites (90%) required over two seconds to load, and the overall average was 8.9 seconds, which far exceeds the best practice recommendation of Google that a webpage load in under three seconds [49]. Dead Link Checker likewise indicated significant problems in regard to links on the evaluated sites, as 22 (71%) had at least one broken link on their homepages; the average was 1.4 inactive links. When auditing entire websites, 25 websites (80.6%) were found to harbor broken links, with an average of 11.2 per website. The greatest number of broken links identified across a site was 133 for the Dawul website. The Yaqeen website did not respond when running the Dead Link Checker; the tool returned only an error message.

Regarding the mobile-friendly test, only the Dawul website did not pass. Three violations of the Google criteria for mobile friendliness were reported: (1) “Content wider than screen causing problem for horizontal scrolling”, (2) “Clickable elements too close together causing touching and tapping difficulties”, and (3) “Text too small to read”.

The manual inspection of each website revealed nearly all of them (97%, *N* = 31) to have neglected to include a search feature; only the website of Osool & Bakheet offered a search bar function. Provision of multilingual features was not good either, as more than half of the websites (56%, *N* = 18) offered only one language for users to interact with the services and information on the site.

## 5. Discussion

This assessment revealed the selected FinTech websites to have significant problems when it comes to accessibility and usability. Despite the evaluation focusing only on landing pages as indicative of the level of web accessibility for visitors [50], no website was found to be fully compliant with guidelines, not even those that consisted of nothing more than a landing page (e.g. Sahem and MAKASSB). These findings underscore the importance of performing evaluations with multiple tools so as to complement their respective limitations and leverage their respective functionalities [51]. For instance, the Emkan and Dinar homepages were found to have errors by both Siteimprove and WAVE, but not by MAUVE++. Conversely, where the Sahem website was indicated to have no errors by WAVE and only two by Siteimprove, MAUVE++ reported 256 violations. In general, MAUVE++ identified a greater number of errors, except in the cases of just six homepages.

When scoring site conformance with WCAG 2.1, errors were summed for each specific level or principle. These associations were not exclusive as one error might relate to multiple SC; for example, the error “Empty heading” ties into both perceivable and operable principles and to both level A and level AA compliance. Thus, as this error occurred 16 times, it added 16 towards the score of each relevant principle and level.

Table 3 lists the 30 different SC for which violations were identified. Eight of those are specific to WCAG 2.1, namely 1.3.6, 1.4.11, 1.4.10, 1.4.13, 1.3.5, 1.3.4, and 2.5.3. Overall, four SC accounted for nearly 52% of identified violations; these were “Info and Relationships”, “Bypass Blocks”, “Identify Purpose”, and “Visual Presentation”. With regard to each level of conformance, 32% of violations corresponded to level A, 22% to level AA, and 46% to level AAA. This finding highlights FinTech websites as currently failing to meet even minimum accessibility requirements. In terms of accessibility principles, the category to which most violations related was perceivable, at 55%, suggesting that it is necessary to give greater regard to supporting the recognition and comprehension of site information and user interface components by disabled users. The principles of operable and robust accounted for similar proportions of violations at 25% and 19%, respectively, while understandable accounted for only 1% of identified violations.

With regard to usability, every one of the evaluated websites had issues; none passed all of the checks employed here. Most websites exhibited average or below average performance, and over half failed to follow best practices concerning page size and load speed as defined by Google [49]. However, only one website was found to have issues in mobile view, specifically content not designed to be displayed on a small screen, too-small text, and elements positioned too close to each other for touchscreen interaction. In fixing these issues, Google recommends CSS elements employ scalable images with appropriate values, webpages use font size scaling with a specified viewport, and that elements such as buttons and navigational links be designed with adequate size and surrounding space [52].

Most of the evaluated sites had issues with broken links, either on the homepage or across the entire site, which impede users in accessing information and navigating pages. Beyond that, broken links are also detrimental to Search Engine Optimization (SEO) due to serving as a signal that a website is dead or outdated, and thereby impacting the site's Google search ranking [53]. In addition, almost all of the examined websites lacked a search feature, further preventing users from quickly finding site content and pages. Finally, a majority of the examined websites only offered their site in one language; given the diversity of innovative FinTech concepts, terminology, and services, lack of multilanguage support may greatly hinder a website's reach among potential users.

Taken together, the present findings indicate that while FinTech websites are generally mobile-friendly, they also exhibit numerous accessibility and usability violations. Moreover, most of the identified errors pertain to the very minimum of accessibility requirements and the perception of information by users. In addition, the websites were generally below average with regard to usability due to excessive page size, the presence of numerous broken links, failure to include a search feature, and providing information in only one language. Most of these accessibility and usability violations are consistent with findings previously reported in the healthcare domain [54–57]. Prior studies found issues with links being empty, color contrast, alternative text for linked images, headings, and keyboard accessibility.

All of the selected FinTech websites in this study concerned financial services in general; none were focused specifically on health information or healthcare financial services in particular. Despite that, the results are not promising and show that people with disabilities have been left behind in terms of the facility of these financial services to support them with healthcare or other needs.

The accessibility and usability of websites constitute essential considerations in the effective delivery of FinTech information and services to users. More work is needed from Saudi FinTech policymakers, designers, and developers in order to ensure that FinTech websites are accessible, usable, and foster a positive user experience for the entire Saudi population, including the 7.1% who are disabled individuals [58]. This practice would follow on the Saudi 2030 vision goals to provide and improve health services to people with different abilities [59], particularly since FinTech innovation has already proven to significantly enhance the sustainable performance of the healthcare sector [60].

## 6. Conclusion

FinTech provides various innovative financial services to people with different abilities, particularly online services. However, this analysis of the accessibility and usability of 32 Saudi FinTech websites revealed substantial room for improvement as not one was fully accessible or perfectly usable. Most accessibility errors related to fundamental requirements such as links and images without alternative text, and most violations to the perceivable principle. Almost all websites were compatible with mobile view, but more than half exhibited inadequate performance with excessive page sizes and load times; moreover, the examined sites harbored many broken links, failed to include a search feature, and presented information in only one language. These findings reveal the difficulties users with disabilities face in accessing FinTech websites and highlight factors that promote a challenging user experience. There remains an essential need to improve these online FinTech services in order to aid disabled individuals and positively affect their opportunities to access services like banking and healthcare systems.

## Figures and Tables

**Figure 1:** Most commonly reported errors (%).

**Table 1:** Reported errors per tool and website ranking.

Website	Mauve++	SiteImprove	WAVE	Total	Avg
Rabet	2004	90	204	2298	766
Positive finance	661	8	11	680	226.67
Sukuk	471	57	33	561	187
Mekyal	335	129	43	507	169
Circlys	313	77	77	467	155.67
Lean	402	31	29	462	154
Scopeer	279	77	93	449	149.67
Rakeez	379	38	29	446	148.67
Dawul	362	49	30	441	147
Hakbah	368	22	46	436	145.33
Money loop	236	88	59	383	127.67
Malaa	254	47	50	351	117
Aseel	266	21	20	307	102.33
Wethaq	276	9	14	299	99.67
Bwatech	265	11	15	291	97
Manafa	223	32	23	278	92.67
Sahem	256	3	0	259	86.33
Raqamyah platform	185	28	34	247	82.33
Osool & Bakheet	196	27	22	245	81.67
Abyan	202	26	15	243	81
Sahlah	178	24	24	226	75.33
Rehan	143	16	31	190	63.33
Emkan	0	85	82	167	55.67
DFN	109	3	1	113	37.67
Afaq	70	26	16	112	37.33
Yaqeen	X	38	57	95	X
Awaed	5	17	33	55	18.33
Buthoor	1	26	15	42	14
Madkhol	2	29	9	40	13.33
Mudaraba	12	11	12	35	11.67
Dinar	0	15	12	27	9
MAKASSB	3	6	5	14	4.67
Total	8456	1166	1144	10766	
			Average	336.34	114.74

**Table 2:** Performance evaluation by Pingdom.

Website	Performance	Page size	Load time (seconds)	Grade
Afaq	64	2.8 MB	6.98	D
Dawul	65	1.7 MB	4.45	D
Positive finance	67	8.5 MB	6.7	D
Wethaq	68	3.4 MB	3.63	D
Circlys	69	2.5 MB	5.71	D
Abyan	69	3.7 MB	8.88	D
Hakbah	70	5.7 MB	9.4	D
Mekyal	70	15.6 MB	1.79	D
Sahlah	72	11.4 MB	8.01	C
Emkan	72	7.2 MB	7.41	C
Mudaraba	72	1.9 MB	9.05	C
Osool & Bakheet	72	2.5 MB	8.17	C
Rabet	73	1.6 MB	2.08	C
Scopeer	73	65.3 MB	26.19	C
Manafa	73	1.1 MB	4.93	C
Raqamyah platform	74	1.7 MB	10.39	C
MAKASSB	74	996.3 KB	91.2	C
Rakeez	75	5.2 MB	3.98	C
Buthoor	76	3.5 MB	3.44	C
Sukuk	77	12.2 MB	7.12	C
Aseel	77	7.82.2 KB	5.45	C
Bwatech	78	1.2 MB	3.21	C
Money loop	79	2.6 MB	4.49	C
Rehan	79	3.5 MB	7.89	C
Lean	80	3.5 MB	1.85	C
DFN	82	3.1 MB	4.4	B
Awaed	82	1.5 MB	2.92	B
Madkhol	92	1.2 MB	2.47	A
Dinar	92	616.3 KB	2.75	A
Sahem	93	463.0 KB	1.33	A
Malaa	95	79.5 MB	12.35	A
Yaqeen	X	X	X	X

**Table 3:** Summary of errors by success criteria.

Success criterion	Description	%
1.3.1	Info and relationships	14.3
2.4.1	Bypass blocks	12.7
1.3.6	Identify purpose	12.68
1.4.8	Visual presentation	12.4
1.4.4	Resize text	6.74
1.1.1	Nontext content	5.07
1.4.11	Nontext contrast	4.97
1.4.3	Contrast (minimum)	4.85
1.4.5	Images of text	4.65
1.4.9	Images of text (no exception)	4.65
1.4.6	Contrast (enhanced)	3.91
2.4.4	Link purpose (in context)	3.32
2.4.7	Focus visible	2.59
1.4.10	Reflow	2.18
2.4.9	Link purpose (link only)	1.93
4.1.2	Name, role, value	1.15
4.1.1	Parsing	0.69
3.3.2	Labels or instructions	0.39
2.4.6	Headings and labels	0.28
1.4.13	Content on hover or focus	0.14
1.3.5	Identify input purpose	0.12
3.1.1	Language of page	0.07
1.4.1	Use of color	0.06
2.1.1	Keyboard	0.04
1.3.4	Orientation	0.03
2.5.3	Label in name	0.03
3.2.2	On input	0.02
2.4.2	Page titled	0.02
2.1.3	Keyboard (no exception)	0.01
2.5.6	Concurrent input mechanisms	0.01

## Data Availability

Data is available upon request.
